# Cytotoxic Activity, Cell Cycle Inhibition, and Apoptosis-Inducing Potential of *Athyrium hohenackerianum* (Lady Fern) with Its Phytochemical Profiling

**DOI:** 10.1155/2022/2055773

**Published:** 2022-06-02

**Authors:** Abdelbaset Mohamed Elasbali, Waleed Abu Al-Soud, Ziad H. Al-Oanzi, Husam Qanash, Bandar Alharbi, Naif K. Binsaleh, Mousa Alreshidi, Mitesh Patel, Mohd Adnan

**Affiliations:** ^1^Clinical Laboratory Science, College of Applied Sciences-Qurayyat, Jouf University, Sakaka, Saudi Arabia; ^2^Department of Pathology, Faculty of Medicine, University of Benghazi, Benghazi, Libya; ^3^Department of Clinical Laboratory Sciences, College of Applied Medical Sciences, Jouf University, Sakaka, Saudi Arabia; ^4^Department of Medical Laboratory Science, College of Applied Medical Sciences, University of Ha'il, Ha'il 55476, Saudi Arabia; ^5^Molecular Diagnostics and Personalized Therapeutics Unit, University of Hail, Ha'il 55476, Saudi Arabia; ^6^Department of Biology, College of Science, University of Hail, Ha'il 2440, Saudi Arabia; ^7^Department of Biotechnology, Parul Institute of Applied Sciences and Centre of Research for Development, Parul University, Vadodara 391760, Gujarat, India

## Abstract

In the present study, we investigated the cytotoxic effects of *Athyrium hohenackerianum* ethanolic extract (AHEE) on the proliferation of breast, lung, and colon cancer cells. The AHEE was tested for its effect on the progression of the cell cycle, followed by induction of apoptosis determination by flow cytometry. Real-time qRT-PCR was also utilized to observe the initiation of apoptosis. In addition, GC-MS was performed in order to identify the active phytochemicals present in the AHEE. A cytotoxic activity with an IC_50_ value of 123.90 *μ*g/mL against HCT-116 colon cancer cells was exhibited by AHEE. Following propidium iodide staining, annexin-V/PI, and clonogenic assays, AHEE treatment results in cell arrest in the S phase, causing an increase in the early and late phases of apoptosis and displaying antiproliferative potential, respectively. The morphological alterations were further monitored using acridine orange/ethidium bromide (AO/EB) staining. When compared with the control cells, features of apoptotic cell death, including nuclear fragmentation, in the AHEE-treated cells were noticed. The apoptosis was also confirmed by detecting the increased expression of *p53* and caspase-3 along with the downregulation of *Bcl-2*. GC-MS analysis revealed that trans-linalool oxide, loliolide, phytol, 4,8,12,16-tetramethylheptadecan-4-olide, and gamma-sitosterol were the major phytochemical constituents. Based on these findings, it can be suggested that AHEE causes cellular death via apoptosis, which should be further explored for the identification of active compounds responsible for these observed effects. Therefore, AHEE can be used in the pharmaceutical development of anticancer agents for cancer therapeutics.

## 1. Introduction

Around the globe, cancer-related deaths are increasing as the incidence of cancer continues to rise [1]. As per the World Health Organization (WHO), colorectal cancer, lung cancer, and breast cancer are the three most frequently diagnosed cancers globally and remain the foremost reason of cancer-related deaths throughout the world [2]. Conventional cancer treatments are still the most common form of treatment, despite being mainly unsuccessful and causing many deaths due to side effects. In contrast, developing new cancer treatments derived from natural sources with fewer side effects has become an exciting field of research [3]. Plants are regarded as a potential repository of novel chemical compounds for cancer research [4]. Many well-known anticancer compounds such as paclitaxel and camptothecin have been reported from plants [5]. India, a biogeographically different region, provides a remarkably rich source of different medicinal plants with anticancer properties [6].

*Athyrium* Roth, commonly known as the lady fern, is one of the cosmopolitan genera in the Athyriaceae family, containing about 300 species distributed around the world. The plants are terrestrial or epilithic, with erect or ascending rhizomes. In diverse areas of the globe, different species of *Athyrium* are used as traditional medicine. There is a tradition that *A. filix-femina* (L.) Roth is utilized with honey for cough treatment in Italy, Province of Salerno, Campania region [7], and its decoction has been used for antiparasitic and antihelminthic purposes [8, 9]. Rhizomes are also used as antiparasitic and antihelminthic agents in Iran as well [10]. *A. pectinatum* (Wall. ex Mett.) T. Moore was used by the Rajasthan Bhils (Indian tribe) as an antihelminthic [11, 12]. Fresh leaf juice of *A. asperum* (Blume) Milde was used as an antihelminthic as well as a carminative in the Mymensingh district of Bangladesh [13]. In Madhya Pradesh (India), *A. falcatum* Bedd. has been used as an antihelminthic [14]. In South India, its roots and fronds were utilized in traditional medicine by the people of the Palani Hills (Western Ghats). As an example, young fronds were consumed as a treatment for cancer and roots were consumed as an antihelminthic [15]. During childbirth, the roots of *A. lanceum* T. Moore are used to relieve pain, particularly breast pain. Besides enhancing milk flow, it is also effective on sores when applied topically [15]. Furthermore, it is used in Malaysia to treat ascariasis, burns, and intestinal fever [16], as well as burns and scalds. The *Athyrium* plant is used to treat sores in New Guinea [17]. In traditional Chinese medicine, *A. multidentatum* has been used as a tranquilizer, antihypertensive, and diuretic [18–20].

*A. hohenackerianum* T. Moore is native to India and Sri Lanka (Figure 1). In India, it is found in different states such as Goa, Gujarat, Jharkhand, Himachal Pradesh Karnataka, Kerala, Maharashtra, Madhya Pradesh, Odisha, Rajasthan, and Tamil Nadu. In India, the rhizome and fronds of *A. hohenackerianum* are used as a decoction for rheumatic pain and as an antihelminthic. The rhizome paste is also used against scorpion stings [21]. To our knowledge, there are no reports regarding any biological activity or phytochemistry of *A. hohenackerianum.* Thus, this study is the initial and first report documenting the anticancer potential and phytoconstituents analysis of *A. hohenackerianum* grown in India.

## 2. Materials and Methods

### 2.1. Collection of Plant Material and Extraction

The collection of *A. hohenackerianum* whole plants was carried out in the South Gujarat region of Gujarat state, India, in September 2020. The voucher specimen (BVBRC042) was deposited at Bapalal Vaidya Botanical Garden, Department of Biosciences, Veer Narmad South Gujarat University, Surat, Gujarat, India. The collected plant material was washed with tap water, and then, deionized water was used to rinse. Thereafter, it was dried under shade at room temperature for 7 days. Upon drying, the samples were ground into powder and were then passed through a sieve that had a mesh size of 20 (sieve size 0.85 mm). 25 g powder of the whole plant of *A. hohenackerianum* was macerated in 85% ethanol in an electric shaker at the room temperature for 6 h. After filtering through Whatman filter paper No. 1, the extract solution was evaporated in a water bath at 60°C for 2 h. A total of 3.40 g of the extract was recovered, which was brown in color, solid in appearance, and bristle in texture.

### 2.2. Cytotoxicity by MTT Assay

The AHEE was tested against human lung (A549), breast (MCF-7), and colon (HCT-116) cancer cells. The National Centre for Cell Science (NCCS), Pune, India, provided cell lines for use in this study. Cancer cell lines were cultured in flasks (25 cm^2^) with 10% fetal bovine serum (FBS) (MP Biomedicals, Germany) in Dulbecco's Modified Eagle's Medium (DMEM) (MP Biomedicals, Germany) and 10,000 U/mL penicillin and 5 mg/mL streptomycin antibiotic solution (Hi-Media, India) at 37°C in a humidified atmosphere with 5% CO_2_. Upon reaching 80% confluence, the cells were seeded at a density of greater than 1 × 10^5^ cells per well in 96-well plates and incubated in the same conditions as above. Trypan Blue (Hi-Media, India) (0.4%) was used to stain the cells, and a hemocytometer was used to determine the viability. Afterward, cells were treated with AHEE at different concentrations (1.56–200 *μ*g/mL) for 48 h. The plate was removed from the incubator, and the media containing AHEE was aspirated. Then, 200 *μ*L of medium containing 10% MTT reagent (MP Biomedicals, Germany) was added to each well to get a final concentration of 0.5 mg/mL, and the plates were incubated for a further 3 h at 37°C in a humidified atmosphere with 5% CO_2_. This was then followed by the removal of the medium and the addition of 100 *μ*L DMSO (Merck, Germany) to dissolve the formazan crystals. Using the ELISA reader (EL10 A, Biobase, China), the absorbance of the amount of formazan crystal was measured at 570 nm and 630 nm. The percentage growth inhibition was calculated after subtracting the background and the blank, and the concentration of the test drug needed to inhibit cell growth by 50% (IC_50_) was calculated from the dose-response curve for the respective cell line. As a positive control, cisplatin was used [22].

### 2.3. Cell Cycle Analysis

The flow cytometer was used to evaluate the cell cycle using propidium iodide (PI) staining. In a six-well culture plate, HCT-116 cells were plated at 5 × 10^4^ cells per 2 mL and incubated in a CO_2_ incubator for 24 h at 37°C. After incubation, the spent medium was aspirated and washed with 1 mL of 1X PBS. Cells were treated with AHEE (IC_50_) concentration in 2 mL of the culture medium and further incubated for 24 h. One well was left blank as untreated, which was considered as a negative control. The floating and attached cells were collected and washed with chilled PBS. Following permeabilization, the cells were fixed for 1 h at 4°C in ice cold 70% ethanol. A staining solution (50 *μ*g/mL PI and 20 *μ*g/mL RNase A in PBS) was then added to the cells for 15 min at 37°C. Samples were mixed well and analyzed with the Cytomics FC500 Flow cytometer, Beckman Coulter, USA [23].

### 2.4. Fluorescent Double Staining with Acridine Orange/Ethidium Bromide (AO/EB)

The cells were plated at a density of 3 × 10^5^ cells/2 mL in 6-well plates and incubated at 37°C for 24 h in a CO_2_ incubator. After aspirating the spent medium, 1 mL of PBS was added. The cells were treated with AHEE (IC_50_) and further incubated for 24 h. For the second time, the medium was removed after incubation and washed in cold PBS. After that, the cells were suspended in 500 *μ*L of AO/EB staining solution (10 *μ*L of acridine orange (2 mg/mL) and 10 *μ*L of ethidium bromide (2 mg/mL) in 1 mL of PBS), mixed thoroughly, and then incubated for 5 min. In the end, cells were washed with PBS bovine serum albumin three times, and images were taken immediately under a fluorescent microscope (XDFL series, Sunny Instruments, China) [24].

### 2.5. Colony Formation Assay

In order to determine the antineoplastic effects on *in vitro* cell proliferation, the clonogenic assay was performed as described previously with minor modifications [25]. In brief, the cells were cultured for 24 h in T-25 tissue culture flasks and exposed to AHEE (IC_50_) for 24 h. Afterward, trypsinization was performed on the cells; the cells were counted and seeded into a 6-well plate (200 cells/2 mL medium per well) and cultured for 8 days. Methanol was used to fix the colonies. Crystal violet (0.4 g/L) was used to stain the colonies, which were photographed, analyzed, and counted using ImageJ (v1.48) software. The formula for calculating the surviving cell fraction was

(1) $$\begin{array}{c} \text{plating efficiency }\left(\text{PE}\right)=\frac{\text{no}.\text{ of cells plated}}{\text{no}.\text{ of colonies counted}}\times 100,\\ \text{surviving fraction }\left(\text{SF}\right)=\frac{\text{PE of treated sample}}{\text{PE of control sample}}. \end{array}$$

### 2.6. Annexin-V Apoptosis Assay

A 6-well plate was seeded with HCT-116 cells at a density of 3 × 10^5^ cells/2 mL and incubated in a CO_2_ incubator at 37°C for 24 h. After removal of the spent medium, 1 mL of PBS was added. The cells were treated with AHEE (IC_50_) in 2 mL of the culture medium and incubated for 12–16 h. An untreated well served as a negative control. At the end of incubation, the medium was removed from all the wells and transferred into 5 mL centrifuge tubes, which were then washed with 500 *μ*L PBS. PBS was removed from the sample, and 200 *μ*L of trypsin-EDTA solution was added and incubated for 3–4 min at 37°C. Afterward, the culture medium was transferred into the respective wells again and cells were harvested into the centrifuge tubes. The tubes were then centrifuged for 5 min at 300 × *g* at 25°C. The supernatant was then removed and washed twice with PBS. The PBS was completely removed, and cells were resuspended in 1X binding buffer at a concentration of 1 × 10^6^ cells/ml. Following this, 100 *μ*L of the solution (1 × 10^5^ cells) was transferred to a 5 mL culture tube and 5 *μ*L of AbFlour 488 Annexin V was added. The cells were gently vortexed and incubated for 15 min at 25°C in the dark. At the end, 2 *μ*L of PI and 400 *μ*L of 1X binding buffer were added to each tube and vortexed gently. Analyses of the samples were carried out by flow cytometry immediately after the addition of PI [26].

### 2.7. Gene Expression Analysis

Tri-Pure Isolation Reagent (Sigma-Aldrich®, India, 11667157001) was used to isolate the cellular RNA according to the manufacturer's instructions, and it was quantified with a nanodrop UV spectrophotometric analyzer (P 300, IMPLEN, USA). The RT-first strand synthesis kit (Qiagen, CA, USA, 330401) was used to reverse transcribe 1 *μ*g of isolated RNA. SYBR green qRT-PCR (Applied Biosystems® 7500 Fast Real-Time PCR machine, CA, USA) was used to measure the gene expression levels relative to control. The 2^−ΔΔCt^ method was used for the analysis, with values expressed as fold changes over the control value. Each primer pair (Table 1) was used separately. The following conditions were used to determine the relative gene expression: reverse transcription was performed at 45°C for 45 minutes as a starting point, initial denaturation at 95°C with 10 min hold, followed by 40 cycles of 95°C for 15 sec, and 60°C for 60 sec [28].

### 2.8. GC-MS Analysis of A. *hohenackerianum* Crude Extract

Shimadzu Nexis GC-2030 equipped with a QP2020 NX mass spectrometer was used for the GC-MS analysis of AHEE. The helium was used as a carrier gas, which flowed at a rate of 1 mL/min. The GC-MS spectral detection method was based on electron ionization energy ionized at 70 eV, a scanning time of 0.2 s, and fragment masses in the range of 40 to 600 m/*z*. A volume of 1 *μ*l and a temperature of 250°C were used for injection. Initially, a temperature of 50°C was set for 3 min in the column oven, then increased by 10°C per min to 280°C, and finally was set to 300°C for 10 min. A comparison of the phytochemicals present in the test samples with a library of authentic compounds maintained by the National Institute of Standards and Technology (NIST) revealed the presence of these compounds based on their mass spectral patterns, retention time (min), peak, area, and height [29].

### 2.9. Statistical Analysis

All experiments were carried out in triplicate. Results are presented as the mean ± SD of the number of experiments performed. The significance of the results was determined among the treatments using one-way ANOVA followed by Tukey's post hoc test and Student's *t*-test at *p* < 0.05. The analyses were carried out using GraphPad Prism 5.0 software.

## 3. Results

### 3.1. Cytotoxic Activity of *A. hohenackerianum* Crude Extract

To determine the cytotoxic activity, various concentrations of AHEE (1.56–200 *μ*g/mL) were applied to A549, MCF-7, and HCT-116 cancer cells and then the IC_50_ values were determined. A dose-response inhibition curve was used to determine the values after 48 hours.  Figure 2 illustrates the dose-response curve of exposure of cancer cell lines to the crude extract. All tested cell lines were sensitive to the crude extract, among which the most sensitive cells were HCT-116 colon cancer cells (IC_50_ = 123.90 *μ*g/mL), more sensitive than MCF-7 breast cancer cells (IC_50_ = 149.92 *μ*g/mL) and lung cancer cells (IC_50_ = 179.74 *μ*g/mL). Therefore, the remaining assays were conducted on the HCT-116 cells. Cisplatin also showed dose-dependent inhibition of HCT-116 colon cancer cells (IC_50_ = 25.95 *μ*g/mL), MCF-7 breast cancer cells (IC_50_ = 36.33 *μ*g/mL), and lung cancer cells (IC_50_ = 43.54 *μ*g/mL).

### 3.2. S Phase Cell Accumulation

A flow cytometry assay was conducted to determine how AHEE affected the cell cycle of HCT-116 cells. An increase was observed in the percentage of cells that are in the *S* phase (40.30 ± 1.35) of the cell cycle in the cells treated with IC_50_ of AHEE with a decline in the percentage of cells in *G*0/*G*1 (33.50 ± 1.19) and G2/M (19.80 ± 1.50) phases in comparison with the untreated control cells. This suggests that the treated cells are arrested in the S phase of the cell cycle (Figure 3).

### 3.3. Morphological Changes in HCT-116 Cells

To explore the morphological alterations caused by AHEE, HCT-116 cells were monitored using AO/EB staining. As compared with the control cells, the features of apoptotic cell death, including nuclear fragmentation, in the AHEE-treated cells were noticed (Figure 4). These results elucidated that the inhibition of AHEE on HCT-116 cell growth is linked with its induction of apoptosis.

### 3.4. Antiproliferative Potential of AHEE

The AHEE was examined for its effect on colony-forming ability in HCT-116 cells. Using AHEE, clonogenic assays were conducted to test the differences between untreated and treated cells in terms of reproductive viability. The colonies formed after 8 days were compared between cancer cells seeded with and without AHEE. A significant reduction in the number of colonies was observed in AHEE (Figure 5).

### 3.5. Quantification of Apoptotic Cell Death of AHEE-Treated Cells

The apoptosis induction by AHEE on HCT-116 cells was further confirmed using the Annexin-V and propidium iodide staining methods. The results of this experiment are shown in Figure 6. After treatment with IC_50_, there was a significant increase from 0.51 ± 0.30% to 9.52 ± 0.92% and 2.80 ± 0.38% to 22.3 ± 1.23% of early and late apoptotic/necrotic cells, respectively.

### 3.6. Expression of Genes Related to Apoptosis

Real-time PCR was used to detect the expression level of the apoptotic genes *p53*, *Bcl-2,* and caspase-3 in HCT-116 cells treated with AHEE. Compared to untreated cells, expression levels of caspase-3 and *p53* were significantly increased, whereas the expression levels of *Bcl-2* were significantly decreased in AHEE-treated cells (Figure 7).

### 3.7. Identification of *A. hohenackerianum* Compounds by GC-MS

The AHEE was analyzed by GC-MS, and different classes of compounds were identified (Table 2). Among the main constituents are butanoic acid, 2,4,6-trimethyloctane, trans-linalool oxide, hexadecane, 1,10-decanediol, loliolide, n-hexadecanoic acid, n-nonadecanol-1, heneicosanoic acid-methyl ester, 10-nonadecanone, phytol, octacosanol, propanoic acid, 2-(benzoylamino)-3-phenyl-m, methyl (Z)-5,11,14,17-eicosatetraenoate, 4,8,12,16-tetramethylheptadecan-4-olide, gamma-sitosterol, hexadecanoic acid-2-hydroxy-1-(hydroxymethyl), octadecanoic acid, 2,3-dihydroxypropyl ester, and androsta-1,4-diene-3,17-dione (Figure 8).

## 4. Discussion

Medicinal plants have been the known source of medicines for the treatment of various ailments since ancient times. People around the globe have implemented the usage of botanicals for millennia. Although angiosperms and other higher plants have been extensively studied for their medicinal and economic value, ferns and fern-allies have been completely overlooked. There is a strong emphasis on its use in Ayurvedic (Sushruta, Charka, and Samhita), Unani, Homeopathic, and other systems of medicine. People use them in the treatment of different kinds of illnesses like burns, colds, ascarid diseases, bleeding due to trauma, and diarrhea [30]. Preliminary screening on different sorts of bioactivities of traditional medicinal ferns has been reported [31–36]. However, no in-depth studies on any biological activities of these plants exist.

*A. hohenackerianum* contains a wide array of phytochemical constituents, making it one of the most valuable medicinal plants [37]. In this study, *A. hohenackerianum* was extracted using ethanol to obtain the largest amount of bioactive phytochemicals. Based on the results of this study, we found that the ethanolic extract of *A. hohenackerianum* conferred high cytotoxic activity on a variety of cancer cells, with good efficacy against human colon cancer cells HCT-116. In addition, we showed that the ethanolic extract of *A. hohenackerianum* arrests the cell cycle at the S phase and specifically induces apoptosis. This fact has been supported by numerous experiments, including labeling with Annexin V-/PI and activation of apoptosis signaling molecules. This study's findings are consistent with a prior study that found other species of *Athyrium* extracts have antiproliferative agents against several cancer cells. It has been reported that *A. multidentatum* shows cytotoxic activity against hepatocellular carcinoma (HepG2 cells) with IC_50_ values of 220 *μ*g/mL and 114 *μ*g/mL after 24 h and 48 h, respectively [38]. It was also reported that *A. multidentatum* crude extract causes cytotoxicity in HL-7702 liver cells with IC_50_ values of 332 *μ*g/mL and 304 *μ*g/mL after 24 h and 48 h, respectively [39]. The butenolide derivative Striatisporolide A of *A. multidentatum* exhibits potent cytotoxic activity against human lung cancer cells (A549) with an IC_50_ of 7.75 *μ*g/mL [39].

To investigate the mechanisms involved in the growth inhibition of HCT-116 cells treated with *A. hohenackerianum*, the cell cycle distribution was analyzed. In the present study, it was found that cells treated with *A. hohenackerianum* accumulated at the S phase of cells, and therefore, this suggests that HCT-116 cells undergo apoptosis since accumulation of cells at this phase is considered a biomarker for DNA damage as well as an indicator of cell death by apoptosis [40]. As part of the confirmation of apoptosis induction, the Annexin-V/PI apoptosis detection assay was used, which is widely used to distinguish both early and late stages of apoptosis [41]. The apoptotic cell death mode of *A. hohenackerianum* was confirmed by a shift toward early and late apoptotic cell populations, suggesting the extract exerted an apoptotic effect. The dual staining of Annexin-V/PI and the cells accumulated in the S phase, as well as the morphological changes that occurred during the cell death evident with AO/EB after treatment with *A. hohenackerianum* crude extract, strongly indicate that the cells are undergoing apoptosis. It is well known that intact plasma membrane integrity can be used as a major indicator of apoptotic cells morphologically [42, 43]. In contrast to apoptosis, necrosis is characterized by a loss of integrity in the cell membrane [42]. The dual AO/EB fluorescent staining method is convenient for detecting changes in cell membranes caused by apoptosis. The AO binds to DNA in intact cells and emits green fluorescence. In damaged cells, EB penetrates the membrane and binds to the DNA and fluorescence of orange-red is emitted [44]. Therefore, AO allows the staining of apoptotic cells as well as live cells, and EB permits the staining of both necrotic and late apoptotic cells.

Furthermore, we also performed a more prolonged clonogenic survival test and found that *A. hohenackerianum* inhibited the survival of HCT-116 cells for a longer period of time. As a result, it should be noted that the crude extract of *A. hohenackerianum* has the potential to be used as a treatment or management for colon cancer, since targeting a cell population that is clonogenic/tumor-initiating/stemlike is believed to be essential for success with cancer therapy.

The apoptotic process is regulated by genes such as *p53*, caspase-3, and *Bcl-2* [45]. A qRT-PCR technique was used to analyze the expression of these apoptotic genes to support the results from the flow cytometry. Compared to the control, treatment with the extracts significantly lowered the antiapoptotic *Bcl-2* gene and significantly increased the apoptotic *Bax* and caspase-3 genes, indicating that *A. hohenackerianum* acts through caspase-dependent apoptotic pathways. It has been reported that a similar event occurred in many studies in which natural product extracts increased the expression of these genes in different human cancer cells, thus causing them to undergo apoptosis [46–49]. Overall, our study confirms that *A. hohenackerianum* induces apoptosis in HCT-116 cancer cells.

The medicinal properties of plant extracts are largely due to the secondary products that act in synergism rather than as a single compound [50–52]. GC/MS is a useful and dependable method for identifying complex plant extracts in an efficient and timely manner [53]. This study identified different classes of phytochemical constituents of *A. hohenackerianum* as having an inhibitory effect on colorectal cancer cells' growth [54], suggesting that these compounds may play a role in the observed activity against HCT-116 colon cancer cells. The natural compound butyric acid is found in food. The anticancer activity of butyric acid has been reported against acute myeloid leukemia, Lewis lung carcinoma cells, and colorectal carcinoma cells [55]. Linalool showed the strongest activity against a broad range of cancers, such as carcinoma of the cervix, stomach, skin, lung, and bone with IC_50_ ranging from 82.3 to 113.6 *μ*g/mL [56]. Phytol is a substance found in chlorophyll and has been shown to be cytoprotective against oxidative stress. The anticancer and immune-enhancing properties of phytol are well-documented. By regulating macrophage function, phytol not only enhances natural killer cells that remove cancer cells but also strengthens immunity. There is evidence that phytol has an anticancer effect against breast, prostate, cervical, colorectal, lung, and skin cancers, with IC_50_ values ranging from 15.51 to 69.67 *μ*M [57]. Gamma-sitosterol is a compound that belongs to the stigmastanes and derivatives family of organic compounds. It has also anticancer effects against several types of cancer including, breast, lung, hepatocellular, and colorectal cancer [58]. Therefore, it can be concluded that the anticancer effects seen in the extract could be due to the presence of these compounds.

## 5. Conclusion

The ethanolic extract of *A. hohenackerianum* inhibited the proliferation of various cancer cells. In particular, we demonstrated that the *A. hohenackerianum* extract inhibits the growth of HCT-116 colon cancer cells by apoptosis by inducing cell arrest in the S phase and causing dose-dependent rises in early and late apoptotic cell populations. Moreover, upregulation of apoptosis gene markers in HCT-116 cells confirmed the initiation of apoptosis by *A. hohenackerianum*. Based on preliminary findings, *A. hohenackerianum* has the potential to be a new natural source of anticolon cancer compound(s) that can trigger apoptotic cell death. However, despite the numerous advantages, toxicity concerns are always present with the variety of plants and can be unsafe for the sensitive populations. Therefore, *in vivo* toxicological assessment is a mandatory requirement and must be done prior to the drug development, which is a limitation in this study. Furthermore, certain assays such as migration assay, angiogenesis assay, and protein expression by Western blotting can also be performed to confirm the efficacy of *A. hohenackerianum* and identify the possible cellular and molecular mechanisms involved in the anticancer activity.

## Figures and Tables

**Figure 1:** *A. hohenackerianum*. (a) Habit, (b) abaxial side of pinnae showing the distribution of sori, (c) close view of sori, (d) and (e) structure of spores under the scanning electron microscope (SEM).

**Figure 2:** Cytotoxic activity of AHEE and standard cisplatin drug against various human cancer cell lines (A549, MCF-7, and HCT-116). (a) Untreated HCT-116 cells. (b) Treated HCT-116 cells with AHEE. (c) Cytotoxicity of cisplatin against A549, MCF-7, and HCT-116. (d) Cytotoxicity of AHEE against A549, MCF-7, and HCT-116. Error bars indicate the SD (standard deviation) of three independent experiments. Significance: ns > 0.05, ^*∗*^ *p* < 0.05, ^*∗∗*^*p* < 0.01, and ^*∗∗∗*^*p* < 0.001.

**Figure 3:** Cell cycle phase distribution in control and treated HCT-116 cells. (a) HCT-116 cell cycle phase distribution of control and after being treated with an IC_50_ concentration of AHEE when analyzed using flow cytometry. (b) Bar graph of the average percentage of cells in different phases of the cell cycle in each treatment and control group. Error bars indicate the SD (standard deviation) of three independent experiments. Significance: ^*∗*^ *p* < 0.05, ^*∗∗*^*p* < 0.01, and ^*∗∗∗*^*p* < 0.001.

**Figure 4:** Dual acridine orange/ethidium bromide staining of HCT-116 cells. (a) Control: untreated cells. (b) Cells treated with an IC_50_ concentration of AHEE. The solid arrow indicates early apoptotic cells, and the dashed arrow indicates late apoptotic cells. The images were taken with a fluorescence microscope at 40x. Live cells are exclusively green, whereas apoptotic cells appear with orange or yellowish-orange nuclei.

**Figure 5:** Clonogenic assay (crystal violet staining) in HCT-116 cells exposed to the IC_50_ concentration of AHEE. (a) Treatment well represents a decrease in the number and size of colonies in comparison to the untreated well and was observed at 10x. (b) A bar graph representing the surviving fraction of HCT-116 cells in the absence and presence of AHEE. Error bars indicate the SD (standard deviation) of three independent experiments. Significance: ^*∗∗∗*^*p* < 0.001.

**Figure 6:** Annexin-V/PI apoptosis assay of treated HCT-116 cells. (a) Distribution of HCT-116 cells without treatment and treatment with IC_50_ concentration of AHEE. (b) A bar graph of cell distribution in control and treated HCT-116 cells, analyzed using flow cytometry. Error bars indicate the SD (standard deviation) of three independent experiments. Significance: ^*∗∗∗*^*p* < 0.001.

**Figure 7:** Gene expression levels in HCT-116 cells treated with the IC_50_ concentration of AHEE. The expression level of apoptosis-related genes was determined via quantitative real-time PCR. *GAPDH* was used as an internal control. Error bars indicate the SD (standard deviation) of three independent experiments. Significance: ^*∗∗*^*p* < 0.01 and ^*∗∗∗*^*p* < 0.001.

**Figure 8:** Chemical structures of the identified compounds in AHEE via GC-MS analysis. (a) Butanoic acid, (b) 2,4,6-trimethyloctane, (c) trans-linalool oxide, (d) hexadecane, (e) 1,10-decanediol, (f) loliolide, (g) n-hexadecanoic acid, (h) n-nonadecanol-1, (i) heneicosanoic acid-methyl ester, (j) 10-nonadecanone, (k) phytol, (l) octacosanol, (m) propanoic acid, 2-(benzoylamino)-3-phenyl-m, (n) methyl (Z)-5,11,14,17-eicosatetraenoate, (o) 4,8,12,16-tetramethylheptadecan-4-olide, (p) gamma-sitosterol, (q) hexadecanoic acid-2-hydroxy-1-(hydroxymethyl), (r) octadecanoic acid, 2,3-dihydroxypropyl ester, and (s) androsta-1,4-diene-3,17-dione.

**Table 1:** List of forward and reverse primers for apoptosis regulatory genes.

Primer	Sequence	Reference
*p53*′	Forward-5′AGAGTCTATAGGCCCACCCC3′ Reverse-5′GCTCGCACGCTAGGATCTGAC3′	[27]

*Bcl-2*	Forward-5′TTCGATCAGGAAGGCTAGAGTT3′ Reverse-5′TCGGTCTCCTAAAAGCAGGC3′	[27]

Caspase-3	Forward-5′TGCGCTGCTCTGCCTTCT3′ Reverse-5′CCATGGGTAGCAGCTCCTTC3′	[27]

GAPDH′	Forward-5′CATGGGGAAGGTGAAGGTCGA3′ Reverse-5′TTGGCTCCCCCCTGCAAATGAG3′	[27]

**Table 2:** Identified phytocompounds from the AHEE via GC-MS.

Compound name	Class	Chemical formula	Molecular weight (g/mol)	RT (min)	Area (%)
Butanoic acid	Fatty ester	C_4_H_8_O_2_	88.11	2.848	0.22
2,4,6-Trimethyloctane	Fatty acyl	C_11_H_24_	156.31	5.781	0.27
trans-Linalool oxide	Terpene alcohol	C_10_H_18_O_2_	170.25	8.870	0.17
Hexadecane	Fatty acyl	C_16_H_34_	226.41	8.935	0.24
1,10-Decanediol	Fatty alcohol	C_10_H_22_O_2_	174.28	9.949	0.26
Loliolide	Monoterpene alkaloid	C_11_H_16_O_3_	196.24	11.127	0.95
*n*-Hexadecanoic acid	Fatty acid	C_16_H_32_O_2_	256.42	12.143	3.26
*n*-Nonadecanol-1	Fatty alcohol	C_19_H_40_O	284.5	12.329	0.35
Heneicosanoic acid, methyl ester	Fatty acid	C_22_H_44_O_2_	340.6	12.476	0.07
10-Nonadecanone	Fatty acyl	C_19_H_38_O	282.5	12.732	0.17
Phytol	Diterpene alcohol	C_20_H_40_O	296.5	12.900	2.04
Octacosanol	Fatty alcohol	C_28_H_58_O	410.76	13.269	0.13
Propanoic acid, 2-(benzoylamino)-3-phenyl-, m	Fatty acid	C_23_H_21_NO_3_	359.4	13.727	1.03
Methyl (Z)-5,11,14,17-eicosatetraenoate	Fatty acid	C_21_H_34_O_2_	318.5	13.877	0.10
4,8,12,16-Tetramethylheptadecan-4-olide	Terpenoid	C_21_H_40_O_2_	324.5	14.021	0.88
Gamma-sitosterol	Phytosterol	C_29_H_52_O_2_	432.7	14.247	4.17
Hexadecanoic acid, 2-hydroxy-1-(hydroxymethyl)	Glycerolipid	C_19_H_38_O_4_	330.5	14.845	2.43
Octadecanoic acid, 2,3-dihydroxypropyl ester	Fatty acid	C_21_H_42_O_4_	358.55	16.293	1.25
Androsta-1,4-diene-3,17-dione	Steroid	C_19_H_24_O_2_	284.39	16.432	0.20

## Data Availability

All data generated or analyzed during this study are included in this article.
